The article "Overexpression of CAPG Is Associated with Poor Prognosis and Immunosuppressive Cell Infiltration in Ovarian Cancer" was retracted in 2023. Reasons: suspected computer-generated content; unreliable results or conclusions; lack of ethics approval or compliance; missing or withdrawn patient consent.

# Overexpression of *CAPG* Is Associated with Poor Prognosis and Immunosuppressive Cell Infiltration in Ovarian Cancer

**DOI:** 10.1155/2022/9719671

**Published:** 2022-02-09

**Authors:** Senwei Jiang, Yuebo Yang, Yu Zhang, Qingjian Ye, Jiao Song, Min Zheng, Xiaomao Li

**Affiliations:** ^1^Department of Gynecology, The Third Affiliated Hospital of Sun Yat-sen University, Guangzhou 510000, China; ^2^Department of Gynecology, Sun Yat-sen University Cancer Center, Guangzhou 510000, China

## Abstract

Historically, immunotherapies have only resulted in a partial response from patients with advanced ovarian cancer, resulting in poor clinical efficacy. A full understanding of immune-related gene expression and immunocyte infiltration in ovarian cancer would be instrumental for the improved implementation of immunotherapy. The Capping Actin Protein, Gelsolin-Like (*CAPG*) gene encodes an actin-regulatory protein, which plays important roles in tumor progression and immune regulation. This study is aimed at identifying the potential therapeutic and prognostic roles of *CAPG* in ovarian cancer. *CAPG* expression and clinical information were investigated in the data collected from TCGA, Oncomine, GEPIA, UALCAN, and Kaplan-Meier plotter. *CAPG* coexpression networks were evaluated by LinkedOmics, GeneMANIA, and NetworkAnalyst. The correlation of *CAPG* with immune infiltrates was analyzed via TIMER, ImmuCellAI, and GEPIA. Our result showed that patients with high tumoral *CAPG* expression had significantly shorter 5-year overall survival. Functional enrichment analysis indicated that *CAPG*-related phenotypes were largely involved in inflammatory response, chemokine and cytokine signaling, cell adhesion, and Toll-like receptor signaling pathways. *CAPG* expression was positively correlated with infiltrating levels of regulatory T cells (Tregs), tumor-associated macrophages (TAMs), and exhausted T cells (Texs) while being negatively correlated with infiltrating levels of natural killer T cells (NKTs) and neutrophils in ovarian cancer. Moreover, the expression of *FOXP3*, *CD25*, *CD127*, *CCR8*, and *TGFβ* in respect to Tregs; *CCL2* and *CD68* in respect to TAM; *CD163*, *VSIG4*, and *MS4A4A* in respect to M2 macrophages; *CD33* and *CD11b* in respect to myeloid-derived suppressor cells (MDSCs); and *PD1*, *CTLA4*, *LAG3*, *TIM3*, *GZMB*, *2B4*, and *TIGIT* in respect to Texs was significantly correlated with *CAPG* expression in ovarian cancer. These findings suggest that *CAPG* may contribute to the immunosuppressive tumor microenvironment in ovarian cancer, leading to an exhausted T cell phenotype and tumor progression. Therefore, *CAPG* can be used as a potential biomarker for determining prognosis and immunotherapy effectiveness in ovarian cancer.

The article "Overexpression of CAPG Is Associated with Poor Prognosis and Immunosuppressive Cell Infiltration in Ovarian Cancer" was retracted in 2023. Reasons: suspected computer-generated content; unreliable results or conclusions; lack of ethics approval or compliance; missing or withdrawn patient consent.

## 1. Introduction

Ovarian cancer (OC) is the most lethal gynecologic malignancy worldwide [1]. Most patients are not diagnosed until they reach advanced stages, contributing to a 5-year overall survival (OS) rate of less than 30% [2]. A combination of surgery and chemotherapy is the classic treatment for ovarian cancer [3]. However, most of stage III–IV patients that have an initial complete response to surgery and chemotherapy will ultimately experience disease progression and resistance to the first-line treatment regimen [4]. Therefore, we urgently need to find novel, more efficient therapies for ovarian cancer.

The primary adjuvant treatment for ovarian cancer has advanced from chemotherapy to targeted molecular therapy [5]. Recently, immunotherapies, such as vaccination, adoptive cellular therapy, and checkpoint inhibitors, have become an attractive therapeutic strategy [6]. Although immune checkpoint blockade (ICB) therapies such as cytotoxic T lymphocyte-associated antigen 4 (CTLA4) and programmed death-1/ligand1 (PD-1/PD-L1) inhibitors showed promising antitumor effects in many cancers, they only exhibited a partial response and poor clinical efficacy in advanced OC [7, 8]. An increasing number of studies have found that the weakness of immunotherapy is dominantly due to the immunosuppressive tumor microenvironment (TME) [9]. Therefore, in order to improve the efficacy of immunotherapies for OC, there is an urgent need for a more comprehensive understanding of immune-related gene expression and immunocyte infiltration in respect to the disease.

The gelsolin protein superfamily is a conserved family of proteins. These proteins have specific roles in actin filament remodeling, cell motility, apoptosis control, phagocytosis regulation, and gene expression regulation [10]. The Capping Actin Protein, Gelsolin-Like (*CAPG*) gene encodes a member of the gelsolin/villin protein superfamily. *CAPG*, also known as Macrophage Capping Protein, reversibly blocks the barbed ends of F-actin filaments in a Ca^2+^ in a phosphoinositide-regulated manner without severing preformed actin filaments [11]. *CAPG* is hypothesized to play a role in regulating cytoplasmic or nuclear structures through interactions with actin, such as cell differentiation, membrane ruffling, and cell motility [12]. Although the function of *CAPG* has not been extensively studied, it has been reported that *CAPG* is upregulated in various malignancies, suggesting its potential role as a tumor driver, particularly contributing to cancer cell invasion and metastasis [13–16]. A previous study shows that bone marrow-derived macrophages of *CAPG* knockout (KO) mice exhibited distinct motility defects [17]. In addition, *CAPG* plays a unique role in receptor-mediated ruffling, phagocytosis, and vesicle rocketing of macrophages [18]. Moreover, a previous study exhibits that *CAPG* has a potential regulating effect in the polarization of tumor-associated macrophages (TAMs) in glioma [19]. *CAPG* has also been reported to be specifically upregulated in Tregs during chronic helminth infection [20]. These findings indicate that *CAPG* may not only function as an oncogene but can prospectively be used as a predictive biomarker for cancer patient prognosis and the immunotherapy efficacy.

The article "Overexpression of CAPG Is Associated with Poor Prognosis and Immunosuppressive Cell Infiltration in Ovarian Cancer" was retracted in 2023. Reasons: suspected computer-generated content; unreliable results or conclusions; lack of ethics approval or compliance; missing or withdrawn patient consent.

Here, we investigated *CAPG* expression in ovarian cancer by utilizing patient data from various public databases. Our results showed that patients with high tumoral *CAPG* expression had significantly shorter 5-year OS. By performing multidimensional database analysis, we evaluated the coexpression and functional networks related to *CAPG* in ovarian cancer. Inflammatory response, chemokine and cytokine signaling, cell adhesion, and Toll-like receptor signaling pathways were enriched in the *CAPG*-related phenotype. Moreover, we investigated the correlation of *CAPG* with tumor-infiltrating immune cells in ovarian cancer microenvironments. We found that *CAPG* expression was positively correlated with infiltrating levels of type 1 Tregs, natural Tregs, induced Tregs, TAMs, and Texs while being negatively correlated with infiltrating levels of NKTs and neutrophils. Furthermore, *CAPG* expression had strong correlations with markers of Tregs, TAMs, MDSCs, and Texs. Our results not only shine a light on the important role of *CAPG* in ovarian cancer but also provide insight into the underlying mechanisms behind *CAPG* and tumor-immune interactions.

## 2. Materials and Methods

### 2.1. TCGA Dataset

The mRNA expression data (379 samples) and clinical information were downloaded from The Cancer Genome Atlas (TCGA) database (https://cancergenome.nih.gov). The following samples were excluded: (1) repeated sequencing results and (2) insufficient survival information. A total of 376 ovarian cancer patients with complete clinical information (i.e., age, sex, primary tumor site, metastatic state at diagnosis, survival time, and survival state) were included in our analysis. Follow-up was started at the time of diagnosis, and OS time was censored at the last date the patient was known to be alive. The expression profiles were extracted from transcriptome RNA High-throughput sequence (HTSeq) data of the ovarian cancer samples. Raw data were processed into Fragments Per Kilobase of transcript per Million mapped reads (FPKM) for further analyses.

The article "Overexpression of CAPG Is Associated with Poor Prognosis and Immunosuppressive Cell Infiltration in Ovarian Cancer" was retracted in 2023. Reasons: suspected computer-generated content; unreliable results or conclusions; lack of ethics approval or compliance; missing or withdrawn patient consent.

### 2.2. Oncomine Database

Oncomine (https://www.oncomine.org) is a cancer microarray database and web-based data-mining platform [21]. Oncomine is often used for validation the expression level of genes in cancers and paired normal tissues in bioinformatic research [22]. Cancer vs. normal analysis was determined according to the following threshold: *p* value of 1*E*-4, fold change of 2.0, and gene rank of top 10%. *CAPG* expression in OC was based on Bonome Ovarian, Yoshihara Ovarian, TCGA Ovarian, and Lu Ovarian datasets.

### 2.3. GEPIA Database

The Gene Expression Profiling Interactive Analysis (GEPIA) database (http://gepia2021.cancer-pku.cn/) is an interactive web that includes tumor and normal samples from TCGA and the GTEx projects [23]. GEPIA was used to generate cancer vs. normal dot plot based on *CAPG* expression in 33 different types of cancer. In addition, the Pearson and Spearman methods were used to determine the gene expression correlation coefficient based on TCGA-OV data. *CAPG* was used for the *y*-axis, and other genes of interest are represented on the *x*-axis.

### 2.4. UALCAN Database

UALCAN (http://ualcan.path.uab.edu) uses TCGA RNA-seq data and Clinical Proteomic Tumor Analysis Consortium (CPTAC) proteomic expression data from different cancer types [24]. UALCAN was used to analyze how the clinical characteristics of ovarian cancer patients were related to *CAPG* gene expression, total protein expression, and phosphoprotein expression. The *t*-test was used to estimate the significance of difference in gene expression levels between groups.

### 2.5. Kaplan-Meier Plotter Database

The Kaplan-Meier plotter (http://kmplot.com/analysis/) is capable to assess the effect of genes (mRNA, miRNA, and protein) on survival in cancers [25]. Sources for the databases include GEO and TCGA. Sources for the analysis include TCGA, GSE9891, GSE65986, GSE63885, GSE26712, and other GEO datasets. The relationship between *CAPG* expression levels and prognosis of ovarian cancer patients was analyzed using the Kaplan-Meier plotter. Patients were split by autoselect best cutoff; the follow-up threshold was 60 months. Excluding biased arrays, 1656 patients were enrolled in overall survival (OS) analysis, and 1435 patients were enrolled in progression-free survival (PFS) analysis.

### 2.6. LinkedOmics Database

LinkedOmics (http://www.linkedomics.org/login.php) is a publicly available portal that includes multiomics data from all 32 TCGA cancer types and 10 CPTAC cancer cohorts [26]. *CAPG* coexpression was analyzed statistically using Pearson's correlation in 303 patients with HiSeq RNA sequencing. Function module of LinkedOmics performs analysis of Gene Ontology, KEGG/Panther pathways, miRNA-target enrichment, and transcription factor-target enrichment by the gene set enrichment analysis (GSEA). The genes were also classified using Gene Ontology (GO) according to biological processes, cellular components, and molecular functions. The rank criterion was false discovery rate (FDR) < 0.05, and 500 simulations were performed; enriched gene sets are postprocessed by affinity propagation methods to reduce redundancy.

The article "Overexpression of CAPG Is Associated with Poor Prognosis and Immunosuppressive Cell Infiltration in Ovarian Cancer" was retracted in 2023. Reasons: suspected computer-generated content; unreliable results or conclusions; lack of ethics approval or compliance; missing or withdrawn patient consent.

### 2.7. GeneMANIA Database

GeneMANIA (http://genemania.org/) finds other genes that are related to a set of input genes [27]. A Gene-Gene Interaction (GGI) network composed of 50 *CAPG* coexpression genes was constructed. These nodes represent genes closely related to *CAPG* in terms of physical interactions, shared protein domains, prediction, colocalization, pathway, coexpression, and genetic interactions.

### 2.8. NetworkAnalyst Database

NetworkAnalyst 3.0 (https://www.networkanalyst.ca/) can create cell type- or tissue-specific protein-protein interaction (PPI) networks, gene regulatory networks, and gene coexpression networks as well as networks for disease, drug, and chemical studies [28]. We use NetworkAnalyst to carry out ovary-specific PPI, TF-gene interactions, and protein–chemical interaction analysis on the *CAPG* coexpression module. *CAPG* coexpression module including the top 100 significant genes was positively and negatively correlated with *CAPG* in TCGA-OV. In these networks, nodes represent individual genes/proteins/chemicals, while the edges which connect nodes correspond to a known, curated interaction between a given pair of nodes.

### 2.9. TIMER Database

TIMER (Tumor IMmune Estimation Resource, http://timer.cistrome.org/) is a comprehensive resource for systematical analysis of immune infiltrates across diverse cancer types [29]. In the outcome module, Cox proportional hazard model's covariates were age, stage, purity, and *CAPG* expression, then present the normalized coefficient of the infiltrate for each model across multiple cancer types in a heat map. Correlations between *CAPG* expression and gene markers of tumor-infiltrating immune cells were explored via correlation modules by Spearman's method; correlations were adjusted by tumor purity and age. *CAPG* was used for the *y*-axis with gene symbols, and related marker genes are represented on the *x*-axis as gene symbols. The gene expression level was displayed with Log2 RSEM.

### 2.10. ImmuCellAI Database

ImmuCellAI (Immune Cell Abundance Identifier, http://bioinfo.life.hust.edu.cn/ImmuCellAI#!/) is a tool to estimate the abundance of 24 immune cells from gene expression dataset including RNA-Seq and microarray data [30]. We use ImmuCellAI to analyze the correlations of *CAPG* expression with immune cell abundance of TCGA-OV datasets. Moreover, immune infiltration score and immune checkpoint blockade (ICB) response prediction of OC patients were assessed by ImmuCellAI.

The article "Overexpression of CAPG Is Associated with Poor Prognosis and Immunosuppressive Cell Infiltration in Ovarian Cancer" was retracted in 2023. Reasons: suspected computer-generated content; unreliable results or conclusions; lack of ethics approval or compliance; missing or withdrawn patient consent.

### 2.11. Statistical Analysis Database

The expression level of the *CAPG* gene in patients with OC was evaluated by using box plots. The cutoff value of *CAPG* expression was selected by ROC curve and Youden's index. The Wilcoxon signed-rank test and logistic regression were performed to analyze the association between clinical features and *CAPG* expression in OC. The Kaplan-Meier analysis was performed to draw survival curves. The univariate Cox analysis is used to screen potential prognostic factors, and multivariate Cox analysis is used to verify the prognostic factors. All statistical analyses were performed using SPSS software (version 19.0) or GraphPad Prism 6; a *p* value less than 0.05 is considered statistically significant.

## 3. Results

### 3.1. The *CAPG* Expression Levels in Different Types of Human Cancers

*CAPG* expressions in tumor and normal tissues of patients across multiple cancer types were analyzed via Oncomine. The results showed that *CAPG* expression was higher in numerous solid tumors when compared to the normal tissues most notably in brain cancer, breast cancer, ovarian cancer, and pancreatic cancer (Figure 1(a)).

To confirm these results, we examined *CAPG* expression across multiple malignancies in the GEPIA database and found that *CAPG* levels were also significantly higher in BRCA (breast invasive carcinoma), GBM (glioblastoma multiforme), OV (ovarian serous cystadenocarcinoma), and PAAD (pancreatic adenocarcinoma) when compared to adjacent normal tissues (Figure 1(b)).

### 3.2. Elevated Expression of *CAPG* in Ovarian Cancer

Although OC is the most lethal gynecologic malignancy worldwide, *CAPG* expression and its potential prognostic impact on OC have not been thoroughly evaluated. To evaluate *CAPG* expression in ovarian cancer, we retrieved data from Oncomine containing multiple ovarian cancer cohorts generated by independent studies. We observed that in all the cohorts analyzed, *CAPG* mRNA level was significantly higher in tumor tissues than in normal tissues (Figure 2(a)). Further subgroup analysis of CPTAC samples in the UALCAN database showed that CAPG protein expression was significantly changed in OC subgroup analysis in respect to disease stage, tumor grade, and age (Figure 2(b)).

### 3.3. Baseline Characteristics of Patients

The RNA-seq data for a total of 376 ovarian cancer patients was acquired from TCGA-OV database. The detailed clinical features are listed in Table S1. Among the 376 participants, 90 were ≤50 years old (24.2%) and 286 were >50 years old (53.7%). All the patients' cancer histological types were serous cystadenocarcinoma (100%). In terms of FIGO stage, 1 patient was stage I (0.3%), 22 were stage II (5.9%), 293 were stage III (77.9%), 57 were stage IV (15.1%), and 3 were not available (0.8%). The 5-year vital status included 146 alive (38.8%) and 230 dead (61.2%).

The article "Overexpression of CAPG Is Associated with Poor Prognosis and Immunosuppressive Cell Infiltration in Ovarian Cancer" was retracted in 2023. Reasons: suspected computer-generated content; unreliable results or conclusions; lack of ethics approval or compliance; missing or withdrawn patient consent.

### 3.4. Correlation between *CAPG* Expression and Clinical Features

The association identified between *CAPG* expression and clinical features in TCGA-OV is summarized in Table 1. ICB response prediction and immune infiltration score were analyzed by ImmuCellAI. *CAPG* expression levels were significantly correlated with 5-year vital status (*p* = 0.028), ICB response prediction (*p* = 0.003), and immune infiltration score (*p* = 6.33*e* − 05). However, *CAPG* expression was not significantly correlated with other clinical features such as FIGO stage, lymphatic invasion, and residual tumor size.

Univariate Cox analysis showed that high *CAPG* expression (HR = 1.359, 95% confidence interval (CI) = 1.025 − 1.801, *p* = 0.033), residual tumor size (HR = 1.294, 95% CI = 1.123 − 1.490,*p* = 3.56*e* − 04), and platinum-free interval (HR = 2.233, 95% CI = 1.907 − 2.615, *p* = 2.07*e* − 23) were unfavorable predictors; however, chemotherapy (HR = 0.276, 95% CI = 0.178 − 0.427, *p* = 8.11*e* − 09) and primary therapy outcomes (HR = 0.321, 95% CI = 0.215 − 0.479, *p* = 2.57*e* − 08) were favorable predictors (Table 2). Further multivariate Cox analysis demonstrated that *CAPG* expression (HR = 1.713, 95% CI = 1.196 − 2.454, *p* = 0.003), residual tumor size (HR = 1.393, 95% CI = 1.141 − 1.700, *p* = 1.11*e* − 03), primary therapy outcomes (HR = 0.430, 95% CI = 0.268 − 0.689, *p* =4.59*e*-04), and platinum-free interval (HR = 2.110, 95% CI = 1.741 − 2.558, *p* = 2.85*e* − 14) were independent prognostic factors for OC.

### 3.5. *CAPG* Expression Is Survival-Associated

Kaplan-Meier survival analysis was used to assess the association between *CAPG* expression and the survival outcomes of TCGA-OV cohorts. Although the two groups' disease-free survival (DFS) showed no significant difference (*n* = 376, *p* = 0.668), the high *CAPG* expression group had significantly shorter overall survival (OS) (*n* = 376, *p* = 0.032) compared to the low expression group (Figure 2(c)). Moreover, we used the Kaplan-Meier plotter database to verify our results. Consistently, in these databases, the high-expression group had significantly shorter OS (*n* = 1657, *p* = 0.0048) and DFS (*n* = 1436, *p* = 0.027) than the low-risk group (Figure 2(d)).

The article "Overexpression of CAPG Is Associated with Poor Prognosis and Immunosuppressive Cell Infiltration in Ovarian Cancer" was retracted in 2023. Reasons: suspected computer-generated content; unreliable results or conclusions; lack of ethics approval or compliance; missing or withdrawn patient consent.

### 3.6. *CAPG* Coexpression Networks in Ovarian Cancer

Gene coexpression reflects common genetic risk factors constituting functional relationships; thus, we examined the coexpression profiles with *CAPG* expression in OC. The function module of LinkedOmics was used to examine *CAPG* coexpression in TCGA-OV cohort. Among all 20032 genes, 2891 genes (dark red dots) showed significant positive correlation with *CAPG*, whereas 3691 genes (dark green dots) showed significant negative correlation (Figure 3(a)). The top 50 significant genes positively and negatively correlated with *CAPG* are shown in the heat map (Figure 3(b)), and a description of the 100 coexpressed genes is detailed in Table S2. The Gene Ontology (GO) slim summary is based upon the 17429 unique Entrez Gene IDs; each biological process, cellular component, and molecular function category is represented by a red, blue, and green bar, respectively (Figure 3(c)).

Overrepresentation Enrichment Analysis (ORA) showed that *CAPG* coexpressed genes participate primarily in biological processes, cellular components, and molecular functions (Figure 3(d)). The top 5 significantly enriched biological processes are positive regulation of cell-cell adhesion, regulation of immune system process, cytokine production, immune response, and cell activation. The top 5 significantly enriched cellular components are nucleoplasm part, catalytic complex, nucleolus, cell surface, and bounding membrane of organelle. The top 5 significantly enriched molecular functions are serine-type peptidase activity, transcription regulator activity, zinc ion binding, RNA binding, and protein domain-specific binding.

### 3.7. GSEA Identifies *CAPG*-Related Signaling Pathways

We performed gene set enrichment analysis (GSEA) on the *CAPG* coexpression datasets to identify Gene Ontology and signaling pathways that were differentially activated in TCGA-OV cohort. Kyoto Encyclopedia of Genes and Genomes (KEGG) pathway analysis showed the top 5 significant enrichment pathways which are antigen processing and presentation, oxidative phosphorylation, lysosome, Th1 and Th2 cell differentiation, and chemokine signaling. Panther pathway analysis showed significantly enriched pathways which are B cell activation, toll receptor signaling, and DNA replication (Figure 4(a)). The gene sets related to cytokine-cytokine receptor interaction, cell adhesion molecules, Th1 and Th2 cell differentiation, oxidative phosphorylation, amino sugar and nucleotide sugar metabolism, and the toll-like receptor signaling pathway showed differential enrichment in the *CAPG* expression phenotype (Figure 4(b)). These results suggest that there is a widespread impact of *CAPG* on the immune regulation, cell mobility, and metabolism.

The article "Overexpression of CAPG Is Associated with Poor Prognosis and Immunosuppressive Cell Infiltration in Ovarian Cancer" was retracted in 2023. Reasons: suspected computer-generated content; unreliable results or conclusions; lack of ethics approval or compliance; missing or withdrawn patient consent.

### 3.8. Regulators of *CAPG* Networks in Ovarian Cancer

To further explore the *CAPG* regulators in respect to OC, we analyzed microRNAs (miRNAs) and transcription factor (TF) enrichment of *CAPG* coexpressed genes by the LinkedOmics database (Table S3). The top 5 most significant miRNAs were MIR-519, MIR-181, MIR-93, MIR-302, and MIR-372. The most enriched TFs were ETS2, PU1, E2F, IRF, NFKB, and YY1.

The protein-protein interaction (PPI) network was assembled based on CAPG coexpressed genes in the TCGA-OV cohort by GeneMANIA. Analysis showed that the 50 most significant coexpressed genes play roles in phagocytosis, leukocyte migration, and the negative regulation of immune system processes (Figure 5(a)). Next, the *CAPG* coexpression network was assembled based on ovary-specific data collected from the DifferentialNet database [31] by NetworkAnalyst (Figure 5(b)). The top 5 hub proteins were DExH-Box Helicase 9 (DHX9), Homeodomain Interacting Protein Kinase 2 (HIPK2), Spi-1 Proto-Oncogene (SPI1), Fibronectin 1 (FN1), and Rac Family Small GTPase 2 (RAC2). Further, a graph of TF-miRNA coregulatory interactions of the CAPG coexpressed genes was constructed based on the RegNetwork database [32] (Figure 5(c)). From this, the top five TFs identified were Spi-1 Proto-Oncogene (SPI1), Myelocytomatosis Oncogene (MYC), MYC-Associated Factor X (MAX), YIN-YANG-1 (YY1), and BCL6 Corepressor (BCOR).

### 3.9. Identifies Potential Target Drugs of *CAPG* Networks

To gain insight into potential target drugs based on our established *CAPG* coexpressed gene network, we examined protein-chemical interactions from the Comparative Toxicogenomics Database (CTD) [33]. Excluding hazardous chemicals, the top 5 drugs were valproic acid, JQ1, tretinoin, vorinostat, and vitamin E (Figure 5(d)). Valproic acid (valproate, VPA) has been tested in the treatment of AIDS and numerous cancers due to its histone-deacetylase-inhibiting effects [34]. It can also resensitize cisplatin-resistant ovarian cancer cells [35]. JQ1 inhibits tumor growth when used in combination with cisplatin, and it suppresses the JAK/STAT signaling pathway in OC [36]. Tretinoin (ATRA), an annexin A2 signaling pathway inhibitor, can inhibit OC proliferation and invasion [37]. Vorinostat (suberoylanilide hydroxamic acid, SAHA) was the first histone deacetylase inhibitor approved by the FDA. It can enhance the activity of the chemotherapy drug, olaparib, by targeting homologous recombination DNA repair in OC [38]. Van Impe et al. reported that a CapG single-domain antibody or nanobody could strongly reduce breast cancer metastasis [39]. Based on these things, these drugs show promising potential as novel therapies against OC via *CAPG* networks that warrants further evaluation.

The article "Overexpression of CAPG Is Associated with Poor Prognosis and Immunosuppressive Cell Infiltration in Ovarian Cancer" was retracted in 2023. Reasons: suspected computer-generated content; unreliable results or conclusions; lack of ethics approval or compliance; missing or withdrawn patient consent.

### 3.10. *CAPG* Expression Is Correlated with Immune Infiltration Level in Ovarian Cancer

Tumor immune phenotypes are independent predictors of the outcome of immunotherapy treatment and OS in ovarian cancer patients [40]. In the ImmuCellAI database, *CAPG* expression also had a significant positive correlation with an abundance of type 1 regulatory T cell (Tr1, *p* = 1.8*e* − 04), natural regulatory T cell (nTreg, *p* = 7*e* − 11), induced regulatory T cell (iTreg, *p* = 4*e* − 05), tumor-associated macrophage (TAM, *p* = 0.0024), and exhausted T (Tex, *p* = 4.8*e* − 06). Meanwhile, *CAPG* expression had a negative correlation with an abundance of natural killer T cell (NKT, *p* = 0.0041) and neutrophil (*p* = 6.6*e* − 04) (Figure 6(a)).

Cox analysis with multiple algorithms (TIMER, CIBERSORT, quanTIseq, XCell, MCP-counter, and EPIC) was used to examine immune infiltration levels across TCGA-OV data, with the covariate being *CAPG* expression. This analysis showed that infiltration levels of naïve B cell, M2 macrophage, EC (endothelial cell), and CAF (cancer-associated fibroblast) were unfavorable predictors, while infiltration levels of CD8+ T cell central memory, CD4+ T memory cell, T follicular helper cell (Tfh), B cell, plasma B cell, M1 macrophage, and plasmacytoid dendritic cell were favorable predictors (Figure 6(b)). Further Kaplan-Meier plots showed that the differences in OS were stratified by both the estimated level of immune cell infiltration and *CAPG* expression level in respect to TCGA-OV cohort. Survival analysis showed that CD8+ T, CD4+ T memory, Tfh, plasma B cell, M1 macrophage, and CAF had a statistically significant positive association with OS while naïve B cell and M2 macrophage had a negative association (Figure 6(c)). These findings strongly suggest that *CAPG* plays a specific role in promoting infiltration of immunosuppressive cells in ovarian cancer.

### 3.11. Correlation between *CAPG* Expression and Immune Marker Genes

Moreover, we focused on the correlation between *CAPG* and immune markers in various immunosuppressive cells present in OC. These immune marker genes included those for T helper 2 cell (Th2), Treg, TAM, M2 macrophage, MDSC, EC, CAF, and Tex. The correlation adjustment in respect to purity or age was done in TIMER (Table 3).

Interestingly, we found that expression of *FOXP3*, *CD25*, *CCR8*, and *TGFβ* in respect to Treg; *CCL2* and *CD68* in respect to TAM; *CD163*, *VSIG4*, and *MS4A4A* in respect to M2 macrophage; *CD33* and *CD11b* in respect to MDSC; and *PD1*, *CTLA4*, *LAG3*, *TIM3*, *GZMB*, *2B4*, and *TIGIT* in respect to Tex was significantly correlated with *CAPG* expression in OC (Figures 7(a)–7(e)). Further GEPIA database analysis showed a correlation between *CAPG* and markers of Treg, TAM, M2 macrophage, MDSC, and Tex which are similar to those in TIMER (Table 4).

The article "Overexpression of CAPG Is Associated with Poor Prognosis and Immunosuppressive Cell Infiltration in Ovarian Cancer" was retracted in 2023. Reasons: suspected computer-generated content; unreliable results or conclusions; lack of ethics approval or compliance; missing or withdrawn patient consent.

Therefore, these results further confirmed that *CAPG* may participate in the recruitment of immunosuppressive cells to ovarian cancer, leading to an exhausted T cell phenotype and eventually tumor progression.

## 4. Discussion

The overexpression of *CAPG* is associated with poorer prognosis in multiple cancers. For instance, *CAPG* was found to be upregulated in bladder cancer and associated with clinical aggressiveness and worse prognosis [16]. Additionally, high *CAPG* levels significantly correlated with shorter relapse-free survival as well as enhanced paclitaxel resistance in breast cancer patients [12]. Although *CAPG* overexpression has been reported in 18/47 (38%) of OC patients [41], *CAPG* expression and its potential prognostic impact on OC have not been thoroughly evaluated. Our study found that *CAPG* gene expression was significantly higher in OC than in normal ovarian tissues and that patients with high *CAPG* expression had significantly shorter OS in TGGA-OV cohort (*n* = 376, *p* = 0.032) and Kaplan-Meier plotter database (*n* = 1657, *p* = 0.0048). Cox analysis confirmed that *CAPG* expression (HR = 1.713, 95% CI = 1.196 − 2.454, *p* = 0.003) was an independent risk factor for OS in OC.

Several studies found that *CAPG* participates in a variety of cell functions and pathways. Gau et al. reported that CAPG was one of the key regulators of actin cytoskeleton/cell adhesion and cell migration associated with the loss of BRCA1 function in OC via quantitative proteomics study [42]. Bahassi et al. investigated *CAPG* involvement in tumor cell motility and cytoskeletal dynamics in a clinically derived human fibrosarcoma cell line [43]. Parikh et al.'s findings suggest that specific motility deficits in macrophages, dendritic cells, and neutrophils render *CAPG*(-/-) mice more susceptible to Listeria infection [17]. Witke et al. reported that the loss of *CAPG* in bone marrow macrophages profoundly inhibits macrophage colony-stimulating factor- (CSF-) stimulated ruffling [18]. Renz et al. noted that increased expression of the CAPG protein triggers an increase in cell motility in invasive breast cancer [44]. To probe the signaling events in controlling abnormal *CAPG* expression, we tested the *CAPG* coexpression network. Consistent with the above studies, we found that *CAPG'*s function enriched in respect to cell-cell adhesion, immune system process, cytokine production, immune response, and cell activation. High *CAPG* expression was associated with cell adhesion, inflammatory response, and chemokine and cytokine signaling pathways.

The article "Overexpression of CAPG Is Associated with Poor Prognosis and Immunosuppressive Cell Infiltration in Ovarian Cancer" was retracted in 2023. Reasons: suspected computer-generated content; unreliable results or conclusions; lack of ethics approval or compliance; missing or withdrawn patient consent.

For mining regulators potentially responsible for *CAPG* dysregulation, we found that CAPG in OC is associated with a network of proteins including DHX9, HIPK2, and Myc family. Puca et al. demonstrated that overexpression of HIPK2 circumvents the blockade of apoptosis in chemoresistant ovarian cancer [45]. Patel et al. found that loss function of DHX9 protected BRCA1-mutant mice against tumorigenesis [46]. Various studies indicate that the Myc family network can be viewed as a functional module which acts to convert environmental signals into specific gene regulatory programs [47]. Yang et al. reported that N-Myc and STAT Interactor (NMI) and CAPG were upregulated in glioblastoma, functioning as an inflammatory response [48]. Sheng et al. showed that cisplatin-mediated miR-145 downregulation increased PD-L1 expression via targeting the c-Myc transcription factor, thereby inducing T cell apoptosis in OC [49]. Jimenez-Sanchez et al. investigated associated immune cell exclusion with the amplification of Myc target genes in treatment-naive OC [50]. Our results, partly in line with the findings in the above studies, showed that *CAPG* participated in cancer progression and immune regulation with genes like Myc. However, the mechanisms behind these interactions require further investigation.

The tumor microenvironment is the noncancerous cells present in and around a tumor having a strong influence on the genomic analysis of tumor samples. These altered signaling pathways in tumor cells help produce a suppressive tumor microenvironment enriched for inhibitory cells, posing a major obstacle for cancer immunity. Tumor cells can secrete cytokines that recruit suppressive cells such as Tregs, immature DCs, MDSCs, TAMs, and CAFs, which make antitumor immune responses more difficult to instigate and sustain [51, 52]. Nelson reported that ovarian tumors are often infiltrated by CD4+ CD25+ FoxP3+ regulatory T cells, which leads to the suppression of antitumor immunity [53]. Cui et al. demonstrated that MDSCs inhibited T cell activation and enhanced ovarian cancer stem cell gene expression, sphere formation, and metastasis [54]. Zhou et al. reported that exosomes released from TAMs transfer miRNAs that induce a Treg/Th17 imbalance and generate an immune-suppressive microenvironment that facilitates OC progression and metastasis [55]. Ji et al. showed that IL-8 secreted from CAFs could stimulate malignant growth and increased OC cisplatin resistance [56]. The above suppressive cells can cause dysfunction in effector T cells, causing a state called “T cell exhaustion.” It is characterized by progressive loss of function, changes in transcriptional profiles, and sustained expression of inhibitory receptors [57]. *PD1*, *CTLA4*, *LAG3*, *TIM3*, and *GZMB* are crucial genes that regulate T cell exhaustion and are associated with inefficient control of tumors [58]. PD1+ TIM3+ CD8+ T cells present all features of functional exhaustion and correlate with poor disease outcome [59]. Our results demonstrate that *CAPG* expression was significantly positively correlated with immunosuppressive cell (Tregs, TAMs, MDSCs, and CAFs) infiltration and T cell exhaustion markers (*PD-1*, *CTLA4*, *TIM3*, *GZMB*, *2B4*, and *TIGIT*). Together, these findings suggest that the *CAPG* plays a crucial role in immune response regulation and T cell exhaustion in OC.

The article "Overexpression of CAPG Is Associated with Poor Prognosis and Immunosuppressive Cell Infiltration in Ovarian Cancer" was retracted in 2023. Reasons: suspected computer-generated content; unreliable results or conclusions; lack of ethics approval or compliance; missing or withdrawn patient consent.

In summary, we showed that high *CAPG* expression is correlated with clinical progression and can be considered an independent risk factor for OS in patients with OC. *CAPG* can regulate a variety of immune-related signaling pathways in OC, which may recruit immunosuppressive cells to create immunosuppressive microenvironment, leading to an exhausted T cell phenotype. The importance of this study is that we discovered that *CAPG* may serve as an important reference indicator of tumor immune cell phenotype and can be used as a prognostic biomarker in OC.

## 5. Conclusions

*CAPG* expression is correlated with clinical progression and considered to be an independent risk factor for OS in patients with ovarian cancer. Cell adhesion, inflammatory responses, chemokine and cytokine signaling pathways, and the toll-like receptor signaling pathway may be pivotal pathways regulated by *CAPG* in ovarian cancer. In addition, increased *CAPG* expression correlates with increased immune infiltration levels in Tex, Tr1, nTregs, iTreg, and TAM. Furthermore, CAPG expression potentially contributes to the regulation of Tex, Treg, TAM, and MDSC. Therefore, *CAPG* likely plays a crucial role in the formation of the immunosuppressive microenvironment and can be used as a prognostic biomarker in ovarian cancer.

## Figures and Tables

**Figure 1:** *CAPG* expression level in cancers. (a) Increased or decreased *CAPG* in datasets of different cancers compared with normal tissues in the Oncomine database. Cell color is determined by the best gene rank percentile for the analyses within the cell. (b) Human *CAPG* expression levels in different tumor types and paired normal tissues from the GEPIA database. Log2 (TPM + 1) scale.

The article "Overexpression of CAPG Is Associated with Poor Prognosis and Immunosuppressive Cell Infiltration in Ovarian Cancer" was retracted in 2023. Reasons: suspected computer-generated content; unreliable results or conclusions; lack of ethics approval or compliance; missing or withdrawn patient consent.

**Figure 2:** CAPG expression level is associated with survival outcome in ovarian cancer. (a) Box plot showing *CAPG* mRNA levels in the Bonome Ovarian, Yoshihara Ovarian, TCGA Ovarian, and Lu Ovarian datasets. (b) CAPG expression in subgroups of patients with ovarian cancer by the UALCAN database. Box-whisker plots showing the protein expression of CAPG in subgroups of OV samples. The central mark is the median; the edges of the box are the 25th and 75th percentiles. ns: not significant; ^∗^*p* < 0.05; ^∗∗^*p* < 0.01; ^∗∗∗^*p* < 0.001. (c–d) Overall survival and disease-free survival in TCGA-OV cohort and Kaplan-Meier plotter database.

**Figure 3:** *CAPG* coexpression genes in HCC (LinkedOmics). (a) The global *CAPG* highly correlated genes identified by Pearson's test in OC. (b) Heat maps showing top 50 genes positively and negatively correlated with *CAPG* in OC. Red indicates positively correlated genes, and blue indicates negatively correlated genes. (c) The Gene Ontology slim summary. (d) Significantly enriched GO annotations of *CAPG* in the OC cohort. BP: biological process; CC: cellular component; MF: molecular function.

**Figure 4:** Enrichment plots from GSEA: (a) significantly enriched KEGG pathway and Panther pathway annotations of CAPG in the OC cohort; (b) gene set enrichment plots of cytokine-cytokine receptor interaction, cell adhesion molecules, Th1 and Th2 cell differentiation, chemokine signaling pathway, oxidative phosphorylation, and amino sugar and nucleotide sugar metabolism with high *CAPG* expression. NES: normalized enrichment score.

**Figure 5:** Significant *CAPG* coexpression networks in OC: (a) protein-protein interaction and function network; (b) ovary-specific protein-protein interaction network; (c) transcription factor-miRNA (TF-miRNA) coregulatory network; (d) protein-chemical interactions network.

**Figure 6:** Correlations of *CAPG* expression with immune infiltration level in OC. (a) Low/high *CAPG* expression with immune cell abundance in TCGA-OV by ImmuCellAI. (b) The multivariable Cox proportional hazard model of *CAPG* expression and immune infiltration level of multiple immune. Red indicates significant positive association, blue indicates significant negative association, and gray denotes a nonsignificant result. (c) Kaplan-Meier plots show the difference of OS stratified by both the immune infiltration level and *CAPG* expression level.

**Figure 7:** Scatterplots of correlations between *CAPG* expression and gene markers of Treg (a), MDSC (b), TAM (c), M2 macrophage (d), and T cell exhaustion (e) in OC.

**Table 1:** Correlations between CAPG expression and clinicopathological features of patients with ovarian cancer.

Clinical characteristics		CAPG low (*n* = 206)	CAPG high (*n* = 170)	*p* value
Race	Asian	6	5	0.972
	Non-Asian	195	159	
Subdivision	Left/right	49	52	0.172
	Bilateral	143	110	
Stage	I + II	13	10	0.76
	III + IV	181	159	
Grade	G1 + G2	26	17	0.384
	G3	172	150	
Lymphatic invasion	Yes	53	47	0.292
	No	21	27	
Venous invasion	Yes	36	27	0.147
	No	17	23	
Residual tumor size	>10 mm	56	40	0.562
	≤10 mm	130	107	
Chemotherapy	Yes	188	158	0.55
	No	18	12	
Targeted molecular therapy	Yes	22	10	0.097
	No	184	160	
Hormone therapy	Yes	20	11	0.256
	No	186	159	
Immunotherapy	Yes	4	6	0.341
	No	202	164	
Radiation therapy	Yes	16	9	0.338
	No	190	161	
Platinum-free interval	≥6 months	111	86	0.533
	<6 months	52	47	
Primary therapy outcomes	SD + PD	142	112	0.372
	CR + PR	24	25	
New tumor event after initial treatment	None/locoregional	82	75	0.399
	Progression/recurrence	124	95	
Vital status (5 years)	Dead	96	98	*0.028*
	Alive	110	71	
ICB response prediction	Response	139	89	*0.003*
	Not response	67	81	
Immune infiltration score	Low	149	89	*6.33E−05*
	High	57	81	

Italic values indicate *p* < 0.05.

The article "Overexpression of CAPG Is Associated with Poor Prognosis and Immunosuppressive Cell Infiltration in Ovarian Cancer" was retracted in 2023. Reasons: suspected computer-generated content; unreliable results or conclusions; lack of ethics approval or compliance; missing or withdrawn patient consent.

**Table 2:** Univariate and multivariate Cox regression analyses of clinical characteristics associated with 5-years OS.

Clinical characteristics	Univariate analysis			Multivariate analysis		
	HR	95% CI	*p* value	HR	95% CI	*p* value
Age (≤50 vs. >50)	1.390	0.971–1.988	0.072	1.391	0.898–2.157	0.140
Race (Asian vs. non-Asian)	1.304	0.482–3.525	0.601			
Subdivision (left/right vs. bilateral)	0.949	0.685–1.314	0.751			
Stage (I + II vs. III + IV)	1.459	0.918–2.321	0.11	0.887	0.573–1.375	0.593
Grade (G1 + G2 vs. G3)	1.263	0.930–1.715	0.135			
Lymphatic invasion (Y vs. N)	1.463	0.845–2.533	0.174			
Venous invasion (Y vs. N)	0.978	0.510–1.878	0.948			
Residual tumor size (>10 mm vs. ≤10 mm)	1.294	1.123–1.490	*3.56E-04*	1.393	1.141–1.700	*1.11E−03*
Chemotherapy (Y vs. N)	0.276	0.178–0.427	*8.11E-09*	—	—	1
Targeted molecular therapy (Y vs. N)	0.573	0.320–1.029	0.062			
Hormone therapy (Y vs. N)	0.821	0.511–1.319	0.416			
Immunotherapy (Y vs. N)	0.473	0.175–1.273	0.138	0.636	0.229–1.769	0.386
Radiation therapy (Y vs. N)	0.721	0.418–1.242	0.238			
Primary therapy outcomes (SD + PD vs. CR + PR)	0.321	0.215–0.479	*2.57E−08*	0.430	0.268–0.689	*4.59E−04*
New tumor event after initial treatment (Y vs. N)	1.150	0.843–1.568	0.377			
Platinum-free interval (≥6 months vs. <6 months)	2.233	1.907–2.615	*2.07E−23*	2.110	1.741–2.558	*2.85E−14*
ICB response prediction (R vs. NR)	0.793	0.589–1.068	0.127	0.743	0.474–1.163	0.194
Infiltration score (low vs. high)	0.820	0.604–1.111	0.201	0.798	0.513–1.241	0.317
*CAPG* expression (high vs. low)	1.359	1.025–1.801	0.033	1.713	1.196–2.454	*3.32E−03*

Abbreviations: HR: hazard ratio; CI: confidence interval; Y: yes; N: no; SD: stable disease; PD: progressive disease; CR: complete response; PR: partial response; R: response; NR: not response. Italic values indicate *p* < 0.05.

The article "Overexpression of CAPG Is Associated with Poor Prognosis and Immunosuppressive Cell Infiltration in Ovarian Cancer" was retracted in 2023. Reasons: suspected computer-generated content; unreliable results or conclusions; lack of ethics approval or compliance; missing or withdrawn patient consent.

**Table 3:** Correlation analysis between *CAPG* and related genes and markers of immune cells in TIMER.

Cell type	Gene markers	Gene symbol	None		Purity		Age	
			Cor	*p*	Cor	*p*	Cor	*p*
Th2	GATA3	GATA3	0.30	*1.05E−07*	0.136	*0.0318*	0.295	*2.60E−07*
	IL4	IL4	0.053	0.362	0.134	*0.035*	0.047	0.426
	IL13	IL13	0.086	0.135	0.102	0.108	0.09	0.126
	CD184	CXCR4	0.014	0.807	−0.006	0.93	0.022	0.706
	CD194	CCR4	0.343	*8.73E−10*	0.183	*3.78E−03*	0.343	*1.58E−09*
	IL5	IL5	−0.067	0.246	−0.037	0.557	−0.071	0.224
Treg	FOXP3	FOXP3	0.38	*7.96E−12*	0.23	*2.48E−04*	0.38	*1.50E−11*
	CD25	IL2RA	0.376	*1.30E−11*	0.205	*1.14E−03*	0.371	*4.83E−11*
	CD127	IL7R	0.342	*9.59E−10*	0.145	*0.0219*	0.338	*2.69E−09*
	CCR8	CCR8	0.325	*7.35E−09*	0.221	4.33*E*−04	0.32	*1.93E−08*
	TGF*β*	TGFB1	0.355	*1.98E−10*	0.132	*0.037*	0.362	*1.54E−10*
TAM	CCL2	CCL2	0.31	*3.40E−08*	0.21	*8.70E−04*	0.32	*2.00E−08*
	CD68	CD68	0.431	*3.98E−15*	0.279	*7.80E−06*	0.439	*2.91E−15*
	IL10	IL10	0.239	*2.72E−05*	0.071	0.267	0.232	*5.71E−05*
M2 macrophage	CD163	CD163	0.341	*1.09E−09*	0.162	*0.01*	0.342	*1.68E−09*
	CD206	MRC1	0.204	*3.43E−04*	0.017	0.789	0.199	*5.82E−04*
	VSIG4	VSIG4	0.348	*4.82E−10*	0.169	*7.69E−03*	0.349	*7.84E−10*
	MS4A4A	MS4A4A	0.339	*1.45E−09*	0.162	*0.01*	0.338	*2.88E−09*
MDSC	CD33	CD33	0.434	*2.44E−15*	0.306	*8.48E−07*	0.439	*2.67E−15*
	CD11b	ITGAM	0.351	*3.35E−10*	0.196	*1.91E−03*	0.357	*3.04E−10*
	CD39	ENTPD1	0.154	*7.35E−03*	0.008	0.904	0.149	0.01
EC	CD31	PECAM1	0.294	*1.88E−07*	0.083	0.189	0.308	*7.02E−08*
	CD34	CD34	0.031	0.592	−0.101	0.113	0.043	0.459
	CD146	MCAM	−0.032	0.575	−0.071	0.263	−0.026	0.655
	SBSN	SBSN	−0.043	0.456	−0.121	0.0575	−0.047	0.424
	Podoplanin	PDPN	0.192	*7.77E−04*	0.022	0.725	0.182	*1.74E−03*
CAF	FAP	FAP	0.323	*8.75E−09*	0.129	*0.0417*	0.318	*2.45E−08*
	CD90	THY1	0.078	0.177	−0.023	0.724	0.079	0.174
	*α*-SMA	ACTA2	0.22	*1.11E−04*	0.031	0.623	0.219	*1.55E−04*
	MFAP5	MFAP5	0.166	*3.74E−03*	0.04	0.526	0.157	*6.89E−03*
Tex	PD1	PDCD1	0.374	*1.69E−11*	0.244	*1.02E−04*	0.378	*2.11E−11*
	CTLA4	CTLA4	0.355	*1.96E−10*	0.207	*1.04E−03*	0.356	*3.22E−10*
	LAG3	LAG3	0.257	*5.74E−06*	0.154	*0.015*	0.258	*7.73E−06*
	TIM3	HAVCR2	0.44	*9.25E−16*	0.292	*2.87E−06*	0.448	*6.58E−16*
	GZMB	GZMB	0.322	*9.38E−09*	0.206	*1.08E−03*	0.326	*1.08E−08*
	2B4	CD244	0.374	*1.75E−11*	0.273	*1.27E−05*	0.369	*6.34E−11*
	TIGIT	TIGIT	0.377	*1.12E−11*	0.219	*4.85E−04*	0.38	*1.47E−11*
	BTLA	BTLA	0.002	0.967	−0.006	0.922	−0.005	0.936
	CD160	CD160	0.014	0.802	0.04	0.529	0.015	0.798

Abbreviations: Cor, *R* value of Spearman's correlation; None, correlation without adjustment; Purity, correlation adjusted by purity; Age, correlation adjusted by age. Italic values indicate *p* < 0.05.

The article "Overexpression of CAPG Is Associated with Poor Prognosis and Immunosuppressive Cell Infiltration in Ovarian Cancer" was retracted in 2023. Reasons: suspected computer-generated content; unreliable results or conclusions; lack of ethics approval or compliance; missing or withdrawn patient consent.

**Table 4:** Correlation analysis between *CAPG* and related genes and immune cell markers in GEPIA.

Cell type	Gene markers	Gene symbol	Cor	*p*
Treg	FOXP3	FOXP3	0.35	*1.10E−13*
	CD25	IL2RA	0.23	*1.10E−06*
	CD127	IL7R	0.24	*3.20E−07*
	CCR8	CCR8	0.21	*1.10E−05*
	TGF*β*	TGFB1	0.25	*1.80E−07*
TAM	CCL2	CCL2	0.24	*3.50E−07*
	CD68	CD68	0.26	*8.00E−08*
	IL10	IL10	0.11	*0.019*
M2 macrophage	CD163	CD163	0.33	*5.90E−12*
	CD206	MRC1	0.10	*7.90E−03*
	VSIG4	VSIG4	0.24	*5.10E−07*
	MS4A4A	MS4A4A	0.22	*3.00E−06*
MDSC	CD33	CD33	0.33	*1.60E−12*
	CD11b	ITGAM	0.19	*6.20E−05*
	CD39	ENTPD1	0.11	*0.019*
Tex	PD1	PDCD1	0.34	*9.30E−13*
	CTLA4	CTLA4	0.28	*4.30E−09*
	LAG3	LAG3	0.20	*2.20E−05*
	TIM3	HAVCR2	0.31	*1.20E−10*
	GZMB	GZMB	0.27	*1.00E−08*
	2B4	CD244	0.24	*4.30E−07*
	TIGIT	TIGIT	0.28	*4.60E−09*
	BTLA	BTLA	0.035	0.47
	CD160	CD160	0.042	0.38

Abbreviations: Cor: *R* value of Spearman's correlation. Italic values indicate *p* < 0.05.

## Data Availability

The authors certify that all the original data in this research could be obtained from a public database. All data generated or analyzed during this study are included in this article.

## Supplementary Materials

Supplementary Materials TABLE S1: clinical characteristics of TCGA-OV patients. TABLE S2: *CAPG* positively/negatively correlated significant genes. TABLE S3: the miRNA target and transcription factor networks of CAPG in OC. Abbreviations: ES: enrichment score; NES: normalized enrichment score; FDR: false discovery rate.

## References

[1] Siegel R. L., Miller K. D., Jemal A. (2020). Cancer statistics, 2020. *CA: A Cancer Journal for Clinicians*.

[2] Lheureux S., Gourley C., Vergote I., Oza A. M. (2019). Epithelial ovarian cancer. *Lancet*.

[3] Yang C., Xia B. R., Zhang Z. C., Zhang Y. J., Lou G., Jin W. L. (2020). Immunotherapy for ovarian cancer: adjuvant, combination, and neoadjuvant. *Frontiers in Immunology*.

[4] De Felice F., Vertechy L., Giudice E. (2021). Evolution of Clinical Trials in Ovarian Cancer Management over the Past 20 Years: Never Settle Down, Always Go Beyond. *Journal of Oncology*.

[5] Beaver J. A., Coleman R. L., Arend R. C. (2019). Advancing drug development in gynecologic malignancies. *Clinical Cancer Research*.

[6] Zhou Y., Chen C. L., Jiang S. W. (2019). Retrospective analysis of the efficacy of adjuvant CIK cell therapy in epithelial ovarian cancer patients who received postoperative chemotherapy. *Oncoimmunology*.

The article "Overexpression of CAPG Is Associated with Poor Prognosis and Immunosuppressive Cell Infiltration in Ovarian Cancer" was retracted in 2023. Reasons: suspected computer-generated content; unreliable results or conclusions; lack of ethics approval or compliance; missing or withdrawn patient consent.

[7] Valero C., Lee M., Hoen D. (2021). Response rates to anti-PD-1 immunotherapy in microsatellite-stable solid tumors with 10 or more mutations per megabase. *JAMA Oncology*.

[8] Ji H., Ren M., Liu T., Sun Y. (2021). Prognostic and immunological significance of CXCR2 in ovarian cancer: a promising target for survival outcome and immunotherapeutic response assessment. *Disease Markers*.

[9] De Felice F., Marchetti C., Palaia I. (2015). Immunotherapy of ovarian cancer: the role of checkpoint inhibitors. *Journal of Immunology Research*.

[10] Silacci P., Mazzolai L., Gauci C., Stergiopulos N., Yin H. L., Hayoz D. (2004). Gelsolin superfamily proteins: key regulators of cellular functions. *Cellular and Molecular Life Sciences*.

[11] Johnston P. A., Yu F. X., Reynolds G. A. (1990). Purification and expression of gCap39. An intracellular and secreted Ca2(+)-dependent actin-binding protein enriched in mononuclear phagocytes. *Journal of Biological Chemistry*.

[12] Chi Y., Xue J., Huang S. (2019). CapG promotes resistance to paclitaxel in breast cancer through transactivation of PIK3R1/P50. *Theranostics*.

[13] Huang S., Chi Y., Qin Y. (2018). CAPG enhances breast cancer metastasis by competing with PRMT5 to modulate STC-1 transcription. *Theranostics*.

[14] Kimura K., Ojima H., Kubota D. (2013). Proteomic identification of the macrophage-capping protein as a protein contributing to the malignant features of hepatocellular carcinoma. *Journal of Proteomics*.

[15] Prescher N., Hansch S., Knobbe-Thomsen C. B., Stuhler K., Poschmann G. (2021). The migration behavior of human glioblastoma cells is influenced by the redox-sensitive human macrophage capping protein CAPG. *Free Radical Biology and Medicine*.

[16] Zhaojie L., Yuchen L., Miao C. (2019). Gelsolin-like actin-capping protein has prognostic value and promotes tumorigenesis and epithelial-mesenchymal transition via the Hippo signaling pathway in human bladder cancer. *Therapeutic Advances in Medical Oncology*.

[17] Parikh S. S., Litherland S. A., Clare-Salzler M. J., Li W., Gulig P. A., Southwick F. S. (2003). CapG(-/-) mice have specific host defense defects that render them more susceptible than CapG(+/+) mice to Listeria monocytogenes infection but not to Salmonella enterica serovar Typhimurium infection. *Infection and Immunity*.

[18] Witke W., Li W., Kwiatkowski D. J., Southwick F. S. (2001). Comparisons of CapG and gelsolin-null macrophages: demonstration of a unique role for CapG in receptor-mediated ruffling, phagocytosis, and vesicle rocketing. *Journal of Cell Biology*.

[19] Wei J., Feng L., Wu L. (2020). Integrated analysis identified CAPG as a prognosis factor correlated with immune infiltrates in lower-grade glioma. *Clinical and Translational Medicine*.

The article "Overexpression of CAPG Is Associated with Poor Prognosis and Immunosuppressive Cell Infiltration in Ovarian Cancer" was retracted in 2023. Reasons: suspected computer-generated content; unreliable results or conclusions; lack of ethics approval or compliance; missing or withdrawn patient consent.

[20] Layland L. E., Mages J., Loddenkemper C. (2010). Pronounced phenotype in activated regulatory T cells during a chronic helminth infection. *Journal of Immunology*.

[21] Rhodes D. R., Yu J., Shanker K. (2004). ONCOMINE: a cancer microarray database and integrated data-mining platform. *Neoplasia*.

[22] Jin C. Y., Du L., Nuerlan A. H., Wang X. L., Yang Y. W., Guo R. (2020). High expression of RRM2 as an independent predictive factor of poor prognosis in patients with lung adenocarcinoma. *Aging (Albany NY)*.

[23] Li C., Tang Z., Zhang W., Ye Z., Liu F. (2021). GEPIA2021: integrating multiple deconvolution-based analysis into GEPIA. *Nucleic Acids Research*.

[24] Chandrashekar D. S., Bashel B., Balasubramanya S. A. H. (2017). *UALCAN: a portal for facilitating tumor subgroup gene expression and survival analyses*. *Neoplasia*.

[25] Gyorffy B. (2021). Survival analysis across the entire transcriptome identifies biomarkers with the highest prognostic power in breast cancer. *Computational and Structural Biotechnology Journal*.

[26] Vasaikar S. V., Straub P., Wang J., Zhang B. (2018). LinkedOmics: analyzing multi-omics data within and across 32 cancer types. *Nucleic Acids Research*.

[27] Warde-Farley D., Donaldson S. L., Comes O. (2010). The GeneMANIA prediction server: biological network integration for gene prioritization and predicting gene function. *Nucleic Acids Research*.

[28] Xia J., Benner M. J., Hancock R. E. (2014). NetworkAnalyst--integrative approaches for protein-protein interaction network analysis and visual exploration. *Nucleic Acids Research*.

[29] Li T., Fu J., Zeng Z. (2020). TIMER2.0 for analysis of tumor-infiltrating immune cells. *Nucleic Acids Research*.

[30] Miao Y. R., Zhang Q., Lei Q. (2020). ImmuCellAI: a unique method for comprehensive T-Cell subsets abundance prediction and its application in cancer immunotherapy. *Advanced Science*.

[31] Basha O., Shpringer R., Argov C. M., Yeger-Lotem E. (2018). The DifferentialNet database of differential protein-protein interactions in human tissues. *Nucleic Acids Research*.

[32] Liu Z. P., Wu C., Miao H., Wu H. (2015). RegNetwork: an integrated database of transcriptional and post-transcriptional regulatory networks in human and mouse. *Database*.

[33] Davis A. P., Grondin C. J., Johnson R. J. (2021). Comparative Toxicogenomics Database (CTD): update 2021. *Nucleic Acids Research*.

[34] Cincarova L., Zdrahal Z., Fajkus J. (2013). New perspectives of valproic acid in clinical practice. *Expert Opinion on Investigational Drugs*.

[35] Lin C. T., Lai H. C., Lee H. Y. (2008). Valproic acid resensitizes cisplatin-resistant ovarian cancer cells. *Cancer Science*.

The article "Overexpression of CAPG Is Associated with Poor Prognosis and Immunosuppressive Cell Infiltration in Ovarian Cancer" was retracted in 2023. Reasons: suspected computer-generated content; unreliable results or conclusions; lack of ethics approval or compliance; missing or withdrawn patient consent.

[36] Bagratuni T., Mavrianou N., Gavalas N. G. (2020). JQ1 inhibits tumour growth in combination with cisplatin and suppresses JAK/STAT signalling pathway in ovarian cancer. *European Journal of Cancer*.

[37] Lokman N. A., Ho R., Gunasegaran K., Bonner W. M., Oehler M. K., Ricciardelli C. (2019). Anti-tumour effects of all-trans retinoid acid on serous ovarian cancer.. *Journal of Experimental and Clinical Cancer Research*.

[38] Konstantinopoulos P. A., Wilson A. J., Saskowski J., Wass E., Khabele D. (2014). Suberoylanilide hydroxamic acid (SAHA) enhances olaparib activity by targeting homologous recombination DNA repair in ovarian cancer. *Gynecologic Oncology*.

[39] Van Impe K., Bethuyne J., Cool S. (2013). A nanobody targeting the F-actin capping protein CapG restrains breast cancer metastasis. *Breast Cancer Research*.

[40] Hornburg M., Desbois M., Lu S. (2021). Single-cell dissection of cellular components and interactions shaping the tumor immune phenotypes in ovarian cancer. *Cancer Cell*.

[41] Glaser J., Neumann M. H., Mei Q. (2014). Macrophage capping protein CapG is a putative oncogene involved in migration and invasiveness in ovarian carcinoma. *BioMed Research International*.

[42] Gau D. M., Lesnock J. L., Hood B. L. (2015). BRCA1 deficiency in ovarian cancer is associated with alteration in expression of several key regulators of cell motility - a proteomics study. *Cell Cycle*.

[43] Bahassi E. M., Karyala S., Tomlinson C. R., Sartor M. A., Medvedovic M., Hennigan R. F. (2004). Critical regulation of genes for tumor cell migration by AP-1. *Clinical & Experimental Metastasis*.

[44] Renz M., Betz B., Niederacher D., Bender H. G., Langowski J. (2008). Invasive breast cancer cells exhibit increased mobility of the actin-binding protein CapG. *International Journal of Cancer*.

[45] Puca R., Nardinocchi L., Pistritto G., D'Orazi G. (2008). Overexpression of HIPK2 circumvents the blockade of apoptosis in chemoresistant ovarian cancer cells. *Gynecologic Oncology*.

[46] Patel P. S., Abraham K. J., Guturi K. K. N. (2021). RNF168 regulates R-loop resolution and genomic stability in BRCA1/2-deficient tumors. *Journal of Clinical Investigation*.

[47] Grandori C., Cowley S. M., James L. P., Eisenman R. N. (2000). The Myc/Max/Mad network and the transcriptional control of cell behavior. *Annual Review of Cell and Developmental Biology*.

[48] Yang Q., Wang R., Wei B. (2018). Candidate biomarkers and molecular mechanism investigation for glioblastoma multiforme utilizing WGCNA. *BioMed Research International*.

[49] Sheng Q., Zhang Y., Wang Z., Ding J., Song Y., Zhao W. (2020). Cisplatin-mediated down-regulation of miR-145 contributes to up-regulation of PD-L1 via the c-Myc transcription factor in cisplatin-resistant ovarian carcinoma cells. *Clinical and Experimental Immunology*.

The article "Overexpression of CAPG Is Associated with Poor Prognosis and Immunosuppressive Cell Infiltration in Ovarian Cancer" was retracted in 2023. Reasons: suspected computer-generated content; unreliable results or conclusions; lack of ethics approval or compliance; missing or withdrawn patient consent.

[50] Jimenez-Sanchez A., Cybulska P., Mager K. L. (2020). Unraveling tumor-immune heterogeneity in advanced ovarian cancer uncovers immunogenic effect of chemotherapy. *Nature Genetics*.

[51] Junttila M. R., de Sauvage F. J. (2013). Influence of tumour micro-environment heterogeneity on therapeutic response. *Nature*.

[52] Richard S. A. (2020). Explicating the pivotal pathogenic, diagnostic, and therapeutic biomarker potentials of myeloid-derived suppressor cells in glioblastoma. *Disease Markers*.

[53] Nelson B. H. (2008). The impact of T-cell immunity on ovarian cancer outcomes. *Immunological Reviews*.

[54] Cui T. X., Kryczek I., Zhao L. (2013). Myeloid-derived suppressor cells enhance stemness of cancer cells by inducing microRNA101 and suppressing the corepressor CtBP2. *Immunity*.

[55] Zhou J., Li X., Wu X. (2018). Exosomes released from tumor-associated macrophages transfer miRNAs that induce a Treg/Th17 cell imbalance in epithelial ovarian cancer. *Cancer Immunology Research*.

[56] Ji Z., Tian W., Gao W., Zang R., Wang H., Yang G. (2021). Cancer-associated fibroblast-derived interleukin-8 promotes ovarian cancer cell stemness and malignancy through the Notch3-mediated signaling. *Frontiers in Cell and Developmental Biology*.

[57] Blank C. U., Haining W. N., Held W. (2019). Defining 'T cell exhaustion. *Nature Reviews: Immunology*.

[58] Wherry E. J., Kurachi M. (2015). Molecular and cellular insights into T cell exhaustion. *Nature Reviews Immunology*.

[59] Fucikova J., Rakova J., Hensler M. (2019). TIM-3 dictates functional orientation of the immune infiltrate in ovarian cancer. *Clinical Cancer Research*.

